The article "Study on Inflammatory Factors in Aneurysmal Perimembranous Ventricular Septal Defect in Congenital Heart Disease" was retracted in 2024. Reasons: signs of a paper mill; suspected computer-generated content; unreliable results or conclusions; concerns about the data.

# Study on Inflammatory Factors in Aneurysmal Perimembranous Ventricular Septal Defect in Congenital Heart Disease

**DOI:** 10.1155/2022/8282624

**Published:** 2022-07-19

**Authors:** Jin Zhou, Ying Liu, Jing Wang, Wei Yan, Yongjian Liu, Litao Chen, Zhixing Du, Qilian Xie

**Affiliations:** ^1^The First Hospital of Hebei Medical University, Shijiazhuang 050031, China; ^2^The Fourth Hospital of Shijiazhuang, Shijiazhuang 050000, China; ^3^Anhui Provincial Children's Hospital, Hefei 230000, China

## Abstract

To detect the expression of inflammatory factors such as interleukin-1*β* (IL-1*β*), interleukin-6 (IL-6), transforming growth factor (TGF-*β*), and tumor necrosis factor (TNF-*α*) in the tumor tissue of ventricular septal defect (VSD) in congenital heart disease and to explore the role of inflammatory response in the formation of aneurysmal perimembranous VSD(APVSD). Children with APVSD of congenital heart disease treated by surgery were selected and divided into true aneurysmal perimembranous group (TAP group) and pseudoaneurysmal perimembranous group (PAP group) according to echocardiography and surgical findings. There were 15 children in the TAP group and 31 in the PAP group. The aneurysmal perimembranous tissue of the two groups of children was collected during the operation. IL-1*β*, IL-6, TGF-*β*, and TNF-*α* were positively expressed in the aneurysmal perimembranous tissue of the two groups, and the expression levels of all inflammatory factors in the PAP group were higher than those in the TAP group, and the difference was statistically significant (*P* < 0.05). The expression levels of IL-1*β*, IL-6, TGF-*β*, and TNF-*α* in the aneurysmal perimembranous tissue of the two groups were negatively correlated with the width of the APVSD breach. IL-1*β*, IL-6, TGF-*β*, and TNF-*α* may be involved in the occurrence and development of APVSD through inflammatory mechanism.

## 1. Introduction

VSD is a common congenital heart disease, and most children with APVSD will have perimembranous aneurysm at birth or shortly after birth [1]. The self-healing rate of APVSD was high, but its mechanism is still unclear. Study had shown that inflammatory responses may be involved in this process [2–4]. In this study, in order to study the role of IL-1*β*, IL-6, TGF-*β*, and TNF-*α* in the formation of APVSD, children with APVSD who were surgically treated in the First Hospital of Hebei Medical University and Anhui Children's Hospital were selected. The expression levels of inflammatory factors in the perimembranous tissue of aneurysm were detected by enzyme-linked immunosorbent assay (ELISA) to explore the role of inflammatory response in the formation of APVSD and the possible mechanism of VSD self-healing.

## 2. Subjects and Methods

### 2.1. Subjects

From July 2009 to June 2013, a total of 46 children with APVSD who received surgical treatment in the First Hospital of Hebei Medical University and Anhui Children's Hospital were selected. The children were divided into TAP group and PAP group. There were 15 children in the TAP group, including 9 men and 6 women, with an average age of 9.3 ± 3.8 years. There were 31 children in the PAP, including 17 men and 14 women, with an average age of 9.3 ± 3.5 years.

Diagnostic criteria for TAP VSD: according to the findings during the operation, the ventricular septum tissue was weak and elongated, forming a pouch-like, protruding to the right ventricular cavity. The pouch had no adhesion to the tricuspid valve and aortic valve, and the periphery of the VSD was composed of membranous tissue and fibrous connective tissue.

Diagnostic criteria for PAP VSD [5, 6]: the shunting orifice of the ventricular defect was adhered to part of the septal valve tissue, local fibrous tissue proliferated, and the right cardiac chamber bulged. There was no real rightward protruding pouch wall.

Exclusion criteria: patients with complex congenital heart disease such as tetralogy of Fallot and other congenital malformations; no heart valve prolapse, pulmonary hypertension; no other heart malformations; no systemic inflammation and immune connective tissue disease.

### 2.2. Methods

1. Philips IEElite advanced cardiac color Doppler ultrasound and Philips IE33 advanced cardiac color Doppler ultrasound systems were used for VSD diagnosis. The frequency of the probe was 3-5 MHz, and they could display the location, size, and the base, width, depth of the perimembranous aneurysm, and the width of the breach in multiple sections, angles, and directions. If there were multiple breaches, it was calculated by the sum of all breach widths
2. Determination of inflammatory factors in aneurysmal perimembranous tissue: aneurysmal perimembranous tissue with a size of 3 mm × 3 mm was taken from the breaches from all children with APVSD during the operation. The tissue was minced and ground sufficiently, and the suspension was collected by centrifugation. The levels of IL-1*β*, IL-6, TGF-*β*, and TNF-*α* were determined by ELISA.

### 2.3. Statistical Analysis

SPSS23.0 was used to process and analyze the data. The measurement data were shown as mean ± standard deviation ($\bar{x}\pm s$), and *t* test was used to compare the means of the two groups, and Spearman correlation analysis was used for correlation. *P* < 0.05 was considered to be statistically significant.

## 3. Results

### 3.1. Clinical Characteristics

There were no significant differences in age, gender, height, weight, body mass index (BMI), and other indicators between the two groups (*P* > 0.05) (Table 1).

### 3.2. Comparison of Inflammatory Factors and Tumor Characteristics between the Two Groups

The expression levels of IL-1*β*, IL-6, TGF-*β*, and TNF-*α* in tissue of PAP group were 10.2 ± 1.5 pg/mL, 31.4 ± 3.4 pg/mL, 64.7 ± 5.8 pg/mL, and 220.3 ± 17.2, which were significantly higher than those in TAP group (9.3 ± 1.4 pg/mL, 29.0 ± 3.4 pg/mL, 58.4 ± 5.2 pg/mL, 197.5 ± 17.5) (*P* < 0.05) (Table 2). However, tumor depth and breach width of TAP group and PAP group were similar.

### 3.3. Correlation of Tumor Depth and Breach Width with the Levels of IL-1*β*, IL-6, TGF-*β*, and TNF-*α* in All APVSD

Correlation analysis showed that the levels of IL-1*β*, IL-6, TGF-*β*, and TNF-*α* in tumor tissue were negatively correlated with the tumor depth (*P* < 0.05), but had no correlation with the breach width (*P* > 0.05) (Table 3).

## 4. Discussion

According to the source and anatomical structure, APVSD of congenital heart disease is divided into true perimembranous aneurysm VSD and pseudoperimembranous aneurysm VSD. The formation of true perimembranous aneurysm is due to the failure to close the fetal membranous ventricular septum in time after birth, the closure of the membranous portion is delayed after birth, and part of the generated membranous portion is continuously pressed under the left ventricular high pressure to form perimembranous aneurysm, leaving the top of the tumor, and the breach causes a left-to-right shunt at the ventricular level. Another common perimembranous aneurysm VSD is the so-called pseudoperimembranous aneurysm, which is a relatively immature fibrous tissue formed by the continuous proliferation and adhesion of the tricuspid valve septum, chordae tendineae, or surrounding tissue [7–9]. Previous study has shown that under the condition of left-to-right shunting of intraventricular blood at the level of VSD chamber, long-term high pressure impacted the inferior membrane defect, causing damage to the perimembranous tissue and the gap of the true perimembranous aneurysm. The damage will stimulate the self-repair of the body tissue. However, the specific repair mechanism is not yet clear. Previous study suggested that the formation of perimembranous aneurysm was related to the remodeling of connective tissue involving metallomatrix proteases (MMPS) [10, 11].

As one of the important members of the IL-1 cytokine family, L-1*β* is an important hyperresponsive proinflammatory cell factor secreted and released mainly by monocytes and macrophages activated under inflammatory conditions, cell damage, or immune responses. It is a key factor in the body's regulation of inflammatory response. On the one hand, it has the function of promoting the repair of damaged tissues; on the other hand, IL-1*β* can play a key role in various acute and chronic inflammatory responses by inducing the release of other inflammatory mediators, proinflammatory cytokines, and chemokines. TNF-*α* is a monokine mainly produced by monocytes and macrophages, which can improve the phagocytic ability of neutrophils and stimulate the secretion of IL-1 and IL-6 by endothelial cells and promote the adhesion of neutrophils and endothelial cells [12, 13]. IL-6 is secreted by activated macrophages, lymphocytes, and epithelial cells and can be induced by IL-1 and TNF-*α*. It is an important mediator of inflammatory response and has both proinflammatory and inhibitory effects. Transforming growth factor-*β* (TGF-*β*) is an important cytokine that regulates cell growth and differentiation and has the effect of regulating the proliferation of fibroblasts, smooth muscle cells, and endothelial cells [14, 15]. Various cells in the body can secrete TGF-*β* in an inactive state, and the cleavage of the protein itself can turn the TGF-*β* complex into an activated TGF-*β*.

Generally, tissues with active cell differentiation often contain high levels of TGF-*β*. TGF-*β* is an important factor regulating cell proliferation and differentiation. It can promote the proliferation and phenotypic transformation of vascular smooth muscle cells, fibroblasts, and other cells and promote the synthesis and secretion of extracellular matrix leading to the thickening of the cardiovascular intima, which is closely related to the occurrence of various cardiovascular diseases. TGF-*β* plays an important role in the occurrence and development of various diseases by inducing the expression of VEGF, promoting endothelial cell proliferation, tissue remodeling, and fibrosis formation [16, 17]. In the early stage of VSD, the contraction of the left ventricle produces a huge pressure to divert blood from the left ventricle to the right ventricle, resulting in an increase in right ventricular preload. Under the impact of high-pressure blood flow, aneurysmal perimembranous tissue will cause myocardial cell damage such as aneurysmal perimembranous tissue, right ventricular endocardium, and chordae tendineae and activate these inflammatory cytokines. TNF-*α* and IL-1*β* further activate MMPS and increase its expression, which are involved in inflammation and tissue proliferation [18, 19]. Our study showed that both the true perimembranous aneurysm VSD and the pseudoperimembranous aneurysm VSD, the above-mentioned inflammatory factors, were expressed in aneurysmal perimembranous tissue, and these inflammatory factors were jointly involved in the proliferation of aneurysmal perimembranous tissue. The persistent proliferative aneurysmal perimembranous tissue eventually closed the gap in the ventricular septum. Therefore, this study may be a more reliable evidence to explain that the perimembranous aneurysm formation was the self-healing tendency of VSD children.

In this study, inflammatory factors were detected in the aneurysmal perimembranous tissue of the TAP and PAP groups. However, by comparison, it was found that the expression intensity of inflammatory factors in the aneurysmal perimembranous tissue of children in PAP group was significantly higher than that of the TAP group. The reason may be related to the histology and location of perimembranous aneurysm in the two groups. The pseudoperimembranous aneurysm is a relatively immature fibrous tissue formed by the continuous proliferation and adhesion of the tricuspid valve septum, chordae tendineae, or surrounding tissue [20]. The left-to-right shunt at the ventricular level had a larger impact force and wider damage area, so the inflammatory response was more severe [21]. Our study also found that the expression levels of inflammatory factors were negatively correlated with the breach width of the perimembranous aneurysm in the TAP and PAP groups. The smaller the breach of the perimembranous aneurysm, the greater the corresponding blood flow resistance and the heavier the tumor tissue damage. This was essentially a reflection of the severity of the injury and the severity of the inflammatory response, which just proved that the pseudoperimembranous aneurysm was an active tissue that can proliferate continuously. The aneurysmal perimembranous tissue was continuously damaged by the impact of blood flow, and the continuous inflammatory response made the aneurysmal perimembranous tissue continue to proliferate [22]. This ability to proliferate allowed the larger defects of the VSD to shrink or even close.

This study confirmed that IL-1*β*, IL-6, TGF-*β*, and TNF-*α* were positively expressed in both the TAP and PAP groups, and the expression levels of all inflammatory factors in the PAP group were higher than those in the TAP group. The expression levels of IL-1*β*, IL-6, TGF-*β*, and TNF-*α* in the perimembranous tissue of aneurysm in both groups were negatively correlated with the width of the APVSD breach IL-1*β*, IL-6, TGF-*β*, and TNF-*α* may be involved in the occurrence and development of APVSD through inflammatory mechanisms. However, due to the small sample size and the large time span of sample selection, the results may be biased. In the future, research will be conducted from the perspective of pathology. In future studies, we will further expand the sample size and do further follow-up work. In addition, we also plan to further examine the regulation of these inflammatory factors in animal models or at the cellular level, and look for the possibility of early diagnosis and targeted therapy.

## 5. Conclusion

IL-1*β*, IL-6, TGF-*β*, and TNF-*α* were positively expressed in the aneurysmal perimembranous tissue of children with APVSD, and their expression levels were negatively correlated with the width and number of APVSD breach. IL-1*β*, IL-6, TGF-*β*, and TNF-*α* may be involved in the occurrence and development of APVSD through inflammatory mechanism.

## Figures and Tables

**Table 1:** Clinical characteristics of children in the two groups.

Groups	Age (years)	Gender (men/women)	Height (cm)	Weight (KG)	BMI (kg/m^2^)
TAP	9.3 ± 3.8	9/6	134.7 ± 18.7	31.3 ± 13.0	16.4 ± 2.1
PAP	9.3 ± 3.5	17/14	135.7 ± 17.7	32.5 ± 12.9	16.9 ± 2.1

**Table 2:** Comparison of inflammatory factors and tumor characteristics between the two groups.

Groups	IL-1*β* (pg/mL)	IL-6 (pg/mL)	TNF-*α* (pg/mL)	TGF-*β* (pg/mL)	Tumor depth (mm)	Breach width (mm)
TAP	9.3 ± 1.4	29.0 ± 3.4	58.4 ± 5.2	197.5 ± 17.5	6.8 ± 1.0	7.0 ± 1.5
PAP	10.2 ± 1.5	31.4 ± 3.4	64.7 ± 5.8	220.3 ± 17.2	6.9 ± 1.0	6.9 ± 1.5
*t*	2.142	2.681	3.706	4.166	0.285	0.246
*P*	0.046	0.038	0.001	<0.001	0.778	0.807

**Table 3:** Correlation of inflammatory factor levels with tumor depth and breach width in children with APVSD.

Tumor characteristics	IL-1*β* (ng/L)		IL-6 (ng/L)		TGF-*β* (pg/mL)		TNF-*α* (pg/mL)	
	*R* value	*P* value	*R* value	*P* value	*R* value	*P* value	*R* value	*P* value
Tumor depth	0.053	0.727	0.149	0.323	0.118	0.434	0.113	0.454
Breach width	-0.595	<0.001	-0.620	<0.001	-0.427	0.003	-0.467	0.001

## Data Availability

The data used to support the findings of this study are included within the article.
